# A Meta-Analysis on Evaluation of Nosocomial Infections Amongst Patients in a Tertiary Care Hospital

This article has been retracted.

**DOI:** 10.1155/2021/4386423

**Published:** 2021-09-29

**Authors:** Baozhi Zhang, Xiao Ling Wu, Ruiping Li

**Affiliations:** The Second Affiliated Hospital Of Guangdong Medical University, Zhanjiang, Guangdong, China

## Abstract

**Background:**

Hospital-acquired infections, also known as nosocomial infections, are one of the many severe outcomes amongst patients in tertiary care hospitals. Hospital-acquired influenza is amongst the most common infection which has affected huge population.

**Objective:**

We have performed a meta-analysis in order to summarize the effects of epidemiology and clinical characteristics in HAI.

**Methods:**

We performed literature review with help of PubMed, Cochrane Library, Embase, Scopus, Web of Science, China National Knowledge Infrastructure (CNKI), The Global Index Medicus (GIM), and other clinical databases till 2021. Many random models were used in order to obtain pooled proportions, mean difference, odds ratio, and CI.

**Results:**

A total of six studies were analyzed, where a total of 491 nosocomial and 4030 nonnosocomial infection cases were reported. The odds ratio of mortality was 0.02 with 95% CI and the risk ration for males was 1.08 with 95% CI.

**Conclusion:**

The proportion of nosocomial infections in cases of influenza was higher in patients admitted in tertiary care hospitals. Thus, a surveillance system for vaccination for all the high-risk patients must be made mandatory.

## 1. Introduction

Nosocomial infections are one of the extensive problems faced by the hospitals at a global level. These nosocomial infections, often termed as hospital-acquired infections (HAIs) or even healthcare-associated infections (HCAI), are a major challenge as it affects large number of patients who are in need of intensive care [1, 2]. The majority of cases of distress and mortality are caused because of the nosocomial infections, where environmental contamination plays a crucial role in the transmission. Human influenza is among the transmissible critical respiratory illness which is spread by influenza A and B virus [3]. The nosocomial infection cases usually occur during the annual pinnacle of the collective influenza activity where the healthcare workforce and the patient visitors (family, relatives, and friends) were identified as the most frequent sources [4]. The most common hospital-acquired infections include the ventilator-associated pneumonia, blood-borne infections, surgical site infections, and urinary tract infections [5–7].

Around 8.7% of the patients in the hospitals fall under the risk of exposure to the nosocomial infections which multiply the complicated conditions such as cancer, surgery, or any cases of organ transplant, thereby surging the mortality rate [8]. In an epidemiological study conducted by WHO in 14 countries across the world, 8.7% cases of nosocomial infection cases were reported. This data ranged from 5.0% cases in North American region to 40% in the Asian subcontinent, Latin America, and Sahara regions of Africa [9].

There is a high range of pathogens which cause nosocomial infections such as *Acinetobacter baumannii*, methicillin-resistant *Staphylococcus aureus* (MRSA), vancomycin-resistant enterococci (VRE), *Clostridium difficile*, and *Pseudomonas aeruginosa* that dwell in the environment for a longer duration [10–12]. There are multiple environmental conditions which influence the presence of microorganisms, where number of people present plays the major role, followed by the level of moisture and material supporting microbial growth [13]. Therefore, for a comprehensive understanding, we have performed meta-analysis on the origin and spread of nosocomial infections in a tertiary care hospital.

## 2. Methodology

### 2.1. Search Strategy

The protocols' preparation was done on the basis of Preferred Reporting Items for Systematic Reviews and Meta-analysis (PRISMA). The outcomes will be outlined on how the articles were filtered and selected for inclusion. The exploration of data was performed using PubMed/MEDLINE (studies from 1997 to May 2021), Web of Science (studies from 2001 to May 2021), The Global Index Medicus (GIM) (studies from 2004 to May 2021), Embase (studies from 1999 to April 2021), Cochrane and China National Knowledge Infrastructure (CNKI), Scopus (studies from 1995–2021), and MeSH library terms and proper usage of keywords.

The combination of keywords used for search were “nosocomial infections,” “hospital-acquired infections (HAIs),” “healthcare-associated infections (HCAI),” “multidrug resistant organism (MDROs),” nosocomial pathogens, environmental contamination, healthcare-acquired infections, and nosocomial bacterial infections. The screening of title and abstract and the entire text review was performed on the prospective studies that were found eligible.

### 2.2. Inclusion Criteria

The inconsistency associated with the inclusion of research works was concluded through discussion. The effort was put in to establish communication with the authors of the papers which were included in the study after filtering. The trials incorporated in the study were based on the types of multiple units with which reported patient data from the entire hospital, discrete clinical wards, or subgroups without sorting a specific disease. The population-related inspection studies which recorded the regularity nosocomial infections and the retrospective or case-control studies with clear and detailed data were also considered. The characteristics of included studies are shown in Table 1.

### 2.3. Exclusion Criteria

Different studies with design structure such as reviews, letters, conference abstracts, case studies, and duplicate publications and the studies missing the crucial data or original data were excluded. Some articles were also removed as they were not accessible even after contacting the authors. The studies which were not written in English were also excluded along with the single reports that consisted of incomplete datasets or guidelines.

### 2.4. Data Analysis and Statistical Assessment

Pooling of data was done by reporting same outcomes and occurrence measures (cumulative incidence and prevalence). Prevalence was here defined as the number of incidences (infections) reported every 100 patient who spent time in hospital for a duration of time and ratio of patients suffering from nosocomial (number of patients suffering from nosocomial infection per 100 patients).

Cumulative incidence (CI) was defined in the analysis as new cases per 100 patients over a duration of time. Data were collected on the basis of prevalence of nosocomial infection, devices linked with infections, ventilator days, incidences of nosocomial infections in ICUs, and CI of SSI, surgical site infection. Random meta-analysis was conducted on all the data's pooled. Forest plot and funnel plot were plotted corresponding with 95% confidence intervals (CIs).

## 3. Results

We analyzed five studies on basis of characteristics of study as mentioned in Table 1.

95% CI was 0.35 (0.29–0.42) which was found for mortality and survival of hospital-acquired influenza, nosocomial infections.

Odds ratio with 95% CI (0.01–0.08) have emphasized that hospital-acquired cases were relatively higher as compared to the CAI in influenza infections of patients in tertiary care hospitals.

HAI cases were higher in comparison to the CAI cases.

Risk ratio was analyzed with 95% CI (0.93–1.26) for identifying the prevalence of nosocomial and nonnosocomial infections in males.

The factor for gender was ruled out for nosocomial infections and males were more prevalent to nonnosocomial infections.

Risk of bias: there was no risk of bias in publication of the studies.

## 4. Discussion and Conclusion

Six studies were involved in the study of evaluating the cases of nosocomial infections in patients admitted in tertiary care hospitals (Figure 1). Influenza cases were studied in this meta-analysis where the hospital-acquired infections (nosocomial) were compared with the community acquired infections (nonnosocomial). An odds ratio (OR) of 0.02 with 95% CI was noted for mortality in cases of nosocomial versus nonnosocomial infections. Risk ratio for cases in males was found to be 1.08 with 95% CI. 95% CI was 0.35 (0.29–0.42) was found for mortality and survival of hospital-acquired influenza, nosocomial infections, as shown in Figure 2 (forest plot), and the funnel plot for the same is shown in Figure 3. Characteristics of study for the patients are shown in Table 2.

Total number of cases reported of nosocomial and nonnosocomial influenza infections of patients in tertiary care hospitals for each study are reported in Table 3. Odds ratio with 95% CI (0.01–0.08) have emphasized that hospital-acquired cases were relatively higher as compared to the CAI in influenza infections of patients in tertiary care hospitals; the forest plot is shown in Figure 4, and the funnel plot showed HAI cases were higher in comparison to the CAI cases are shown in Figure 5.

Number of males reporting influenza cases in nosocomial and nonnosocomial category in tertiary care hospitals are shown in Table 4; the risk ratio was analyzed with 95% CI (0.93–1.26) for identifying the prevalence of nosocomial and nonnosocomial infections in males, and its forest plot is shown in Figure 6, while the funnel plot on the risk ratio of the number of males affected by nosocomial infections in tertiary care hospital, and its prevalence in Figure 7.

As the ratio of hospital-acquired infections (nosocomial) is increasing in patients admitted in tertiary care hospitals, hence, a strict surveillance must be enforced for higher risk patients. In cases of diseases such as influenza which has high affinity in nosocomial infections, a system of vaccination must be implied for admissions.

## Figures and Tables

**Figure 1:** PRISMA study for the learning process.

**Figure 2:** Forest plot on mortality and survival rates in nosocomial infections and the risk difference with 95% CI was noted.

**Figure 3:** Funnel plot on mortality and survival rates in nosocomial infections was analyzed in both survival cases and mortality.

**Figure 4:** Forest plot of nosocomial versus nonnosocomial infections (for both HAI and CAI cases).

**Figure 5:** Funnel plot on the odds ratio of incidences of nosocomial versus no-nosocomial infections (for both HAI and CAI cases).

**Figure 6:** Forest plot on risk ratio of gender-based effect of nosocomial infections in tertiary care hospitals.

**Figure 7:** Funnel plot on risk ratio of number of males affected by nosocomial infections in tertiary care hospital and its prevalence.

**Table 1:** Characteristics of included studies.

Characteristics	[14]	[15]	[16]	[17]	[18]	[19]
Study design	Case control	Case	Cross sectional	Cross sectional	Cross sectional	Cross sectional
Sample size	382	1722	208	292	860	2421
Mean age of patients (HAI) nosocomial	62	N/A	79.1	79	82	53.47
Mean age of patients (CAI)	60.4	N/A	64.8	76	47	48.86
Gender	46.5% female	43.1% female	50% female	35.7% female	54.38% female	42.88% female
Duration of study	2017-2018	2010/2011–2015/2016	2016/12–2017/02	2017	2020	2009–2015
Country	United States	Spain	France	Australia	France	Spain
Study quality	7	8	7	6	6	7

**Table 2:** Cases of mortality and survival in hospital-acquired influenza, nosocomial infections.

S. No.	Characteristics	[15]	[16]	[16]	[17]	[18]	[19]
1.	Mortality	4	18	N/A	2	N/A	76
2.	Survived	33	78	N/A	26	N/A	148
3.	Total nosocomial	37	96	49	28	57	224

**Table 3:** Total number of cases reported of nosocomial and nonnosocomial influenza infections of patients in tertiary care hospitals.

Characteristics	[14]	[15]	[16]	[17]	[18]	[19]
HAI	37	96	49	28	57	224
CAI	75	1626	159	264	803	1103
Total	112	1722	208	292	860	1327

HAI, hospital-acquired infection; CAI, community-acquired infection. The above table mentions the events recorded for both nosocomial and nonnosocomial influenza infection cases.

**Table 4:** Gender-based analysis; number of males reporting influenza cases in nosocomial and nonnosocomial category in tertiary care hospitals.

Characteristics	[14]	[15]	[16]	[17]	[18]	[19]
HAI	23	53	17	18	31	142
N (HAI)	37	96	49	28	57	224
COI	35	926	87	122	392	626
N (CAI)	74	1626	159	264	803	1103

HAI, hospital-acquired infection; CAI, community-acquired infection; *N* = number.

## Data Availability

The data that support the findings of this study are available from the corresponding author upon reasonable request.

## Abbreviations:

CI: Confidence interval
SSI: Surgical site infection
CLABSI: Central line-associated bloodstream infection
HAI: Hospital-acquired infection
CAI: Community-acquired infection
VAP: Ventilator-associated pneumonia
CVC: Central venous catheter
ICU: Intensive care unit
OR: Odds ratio
RR: Risk Ratio
HR: Hazard ratio.
